# Research on the Oxidative Stress Response of Human Body Caused by Different Nutritional Supplements and the Improvement Effect of Exercise

**DOI:** 10.1155/2022/1355254

**Published:** 2022-06-08

**Authors:** Shanjia Zhang

**Affiliations:** College of P.E., Xuchang University, Xuchang 461000, Henan, China

## Abstract

This paper combines experimental and observational research to investigate the effect of various nutritional supplements on human oxidative stress response and exercise. Furthermore, this paper investigates the neural pathways involved in motor regulation in the cerebral cortex, striatum, and midbrain. The midbrain is an important site for regulating direct and indirect pathways, as well as motor control. Simultaneously, this paper provides a theoretical foundation as well as experimental value for further understanding the effects of iron deficiency and iron overload on brain iron storage in young adults. Furthermore, this paper provides guidance and a scientific foundation for reasonable exercise for adolescents with iron overload and iron deficiency, as well as an experimental foundation and theoretical support for the development of iron fortifier supplementation and sports foods for special populations. The experimental results validate the method's efficacy.

## 1. Introduction

Exercise-induced fatigue refers to the inability of the body to maintain its function at a certain level or to maintain a predetermined exercise intensity in the physiological process of the body. Taking certain recovery measures after exercise can supplement the consumed energy or even achieve excessive recovery, which will not only help fatigue recovery but also achieve the purpose of maintaining health through exercise. Low-intensity exercise increases free radicals in the body but increases levels of antioxidants and mitochondrial enzymes. It is mainly due to the physiological adaptation caused by low-intensity exercise, which reduces oxidative stress, so low-intensity can regulate the function of cells, which is a beneficial stress. During moderate-intensity exercise, free radical levels rise and long-term moderate-intensity exercise increases antioxidant enzyme activity. During high-intensity intense exercise, the concentration of serum antioxidant enzymes increases, and the content of free radicals also greatly increases, resulting in mitochondrial dysfunction, oxidative damage, and neurotrophic protein decline. Increased peroxidative free radicals and fast purine breakdown cause large quantities of oxygen free radicals in the body, disrupting the antioxidant system's homeostasis. This causes fatigue, muscle discomfort, muscle fiber rupture, and decreased immunological function during and after exercise. During high-intensity exercise, antioxidant enzymes may be selectively activated depending on tissue oxidative stress and enzyme intrinsic activity. The greater the intensity, the longer the duration of exercise, and the more obvious the increase in the activities of skeletal muscle SOD (superoxide dismutase) and GSH-Px (glutathione peroxidase).

The main nutrients in the diet during exercise are carbohydrates. In endurance sports, the supply of sugar in the body is the limiting factor for performance improvement. During exercise, the appearance of fatigue and the decline in the level of exercise performance are closely related to the decline in the availability of carbohydrates in the body [1]. Therefore, athletes supplementing sugar-containing nutrients in time before, during, and after long-term strenuous exercise can help maintain blood sugar levels during exercise, increase muscle glycogen reserves, improve exercise endurance, and maintain physical health. There are studies that suggest increasing protein requirements for athletes. The main reasons include repairing exercise-induced damage to muscle fibers, protein as a source of energy during exercise, and the need for additional protein to increase lean body mass [2]. If protein requirements increase, the degree of increase may depend on gender, exercise type, intensity, duration, etc. [3].

Micronutrients play an important role in producing energy and Hb, maintaining bone health, ensuring immune function, and protecting body tissues from oxidative damage. Also, micronutrients help synthesize and repair muscle tissue after exercise. In theory, exercise can increase or change the need for vitamins and minerals under different circumstances. However, exercise inhibits many metabolic mechanisms that require micronutrients, so exercise training may produce biochemical adaptations in muscles that increase micronutrient requirements. In addition to this, exercise may prompt micronutrient shifts and increase micronutrient losses. This work studies the influence of nutritional supplements on human oxidative stress response and exercise, providing a theoretical reference for exercise enhancement and nutritional supplementation.

## 2. Related Work

Literature [4] used the potassium ferricyanide method, methyl violet method, pyrogallol auto-oxidation method, and DMPD method to detect the effects of vitamin C and vitamin E alone and combined with the various physiological activities of vitamin C and vitamin E. With the reducing power and the scavenging ability of DMPD + free radicals, hydroxyl free radicals, and superoxide ions, it was found that vitamin C is better than vitamin E in terms of reducing ability and free radical scavenging ability, the combined effect of the two is stronger than the single effect, and the combined effect of the two is on AAPH. The resulting protein oxidative damage has a protective effect. The reducing ability of a substance is an important manifestation of its potential antioxidant activity, and the strength of the reducing ability shows the strength of the antioxidant activity of the substance to a certain extent. C is related to hydrophilic antioxidants, and OH and O2 are two common oxygen free radicals. The combination of vitamin C and vitamin E can effectively clear OH and O2, and the effect is better than that of a single action activity [5].

Literature [6] after the mice in the experimental group were given low, medium, and high doses of Lycium barbarum polysaccharide and the same amount of normal saline was given to the control group for weight-bearing swimming, the weight-bearing swimming time, SOD activity, MDA value, liver glycogen, and muscle were measured. Glycogen, serum urea nitrogen, lactic acid content, and other indicators, it was found that the weight-bearing swimming time of the mice in the wolfberry polysaccharide group was significantly prolonged, the SOD activity increased, the MDA content decreased, the liver glycogen and muscle glycogen content increased, and the serum urea nitrogen and lactic acid content decreased, indicating that Lycium barbarum polysaccharide has antifatigue activity. Lycium barbarum is the dried fruit of the Solanaceae plant Ningxia Lycium barbarum, and its pharmacological effects are to nourish the kidney and nourish yin, cure deficiency, and quench thirst. Lycium barbarum polysaccharide is the main active ingredient of Lycium barbarum. By improving SOD activity in mice, reducing MDA content, reducing the accumulation of free radicals in the body, and accelerating the clearance of lipid peroxides, Lycium barbarum polysaccharide can improve exercise capacity and delay exercise. Fatigue has a positive effect on maintaining the reserves of liver glycogen and muscle glycogen, improving the body's exercise load capacity, accelerating the clearance of metabolites, and slowing the occurrence of exercise-induced fatigue [7]. In literature [8], the mice in the experimental group were given total flavonoids of Rubescens by gavage and the control group was supplemented with the same amount of purified water. After swimming to exhaustion, the levels of malondialdehyde (MDA) and MDA in the serum and skeletal muscle of the mice were determined. Blood lactate content, superoxide dismutase (SOD), glutathione peroxidase (GSH-Px), catalase (CAT), and lactate dehydrogenase (LDH) activity in skeletal muscle, it was found that the mice in the experimental group had higher levels of lactate dehydrogenase (LDH). The activity of various antioxidant enzymes was significantly enhanced, and the onset of exercise-induced fatigue was delayed. It shows that the total flavonoids of Rubescens can effectively inhibit the generation of free radicals in the serum and gastrocnemius muscle of mice because the total flavonoids of Rubescens can improve the scavenging efficiency of oxygen free radicals in the body, increase the activity of corresponding antioxidant enzymes, and reduce MDA. It is proved that the total flavonoids of Rubescensica can enhance the body's antioxidant capacity, and it is an antifatigue sports supplement with high potential nutritional value [9]. Literature [10] by gavage high and low doses of Agaricus ethanol extract in the experimental group, normal group, exercise-induced fatigue model, and ginsenoside group, and after treadmill exhaustive exercise, myocardial MDA, SOD, GSH-Px, MDA, SOD, GSH-Px, MDA, SOD, GSH-Px, MDA, SOD, GSH-Px, MDA, SOD, GSH-Px, MDA, SOD, MDA, SOD, GSH-Px, MDA, SOD, GSH-Px, MDA, SOD, GSH-Px, and MDA levels were measured. T-AOC content, it was found that the exhaustive exercise time increased, the myocardial MDA content decreased, and the SOD, GSH-Px, and TAOC activities increased in the drug intervention group, indicating that the alcoholic extract of Agrimony spp. oxidative capacity, which may alleviate the myocardial oxidative stress injury of exercise-induced fatigue by improving the myocardial antioxidant capacity and reducing lipid peroxidation in exercise-induced fatigue rats. Ginsenosides have been confirmed by research to be effective antioxidants. The experimental results confirmed that Agrimony grass extracts and ginsenosides have similar effects. The antioxidant activity of Agrimony grass has been affirmed. The main antioxidant components are flavonoids, tannins, and polyphenols class ingredients. Agrimony ethanol extract has a certain research value as a natural antioxidant [11].

The way of iron supplementation for athletes should be mainly diet. The iron provided in the diet is mainly nonheme iron, which generally accounts for more than 80% of the iron content of the food. Nonheme iron mainly exists in vegetables, fruits, and cereal crops, and its absorption rate is greatly affected by dietary components, dietary habits, and iron storage in the body, and its absorption and availability are generally 3%–8% [12]. Heme iron is mainly found in animal meat, and maintaining or increasing the intake of animal protein can provide athletes with abundant heme iron. Athletes should follow correct dietary habits when supplementing with dietary iron [13]. When the diet cannot provide sufficient iron, it should be considered to supplement iron in the form of iron preparations. The main components of iron preparations are inorganic iron and organic iron, which can be divided into heme iron and nonheme iron according to their existing forms in the human body. There are two categories [14]. Research results show that heme iron and organic iron are the best forms of iron supplementation for athletes [15]. Heme iron and organic iron have the advantages of easy absorption, less dosage, no or less side effects, and fewer affected factors. They are currently the best iron preparations for the prevention of iron deficiency and IDA in the sports industry. Antioxidants can significantly improve iron absorption [16]. It is worth noting that athletes should strengthen the monitoring of iron metabolism indicators when using iron preparations. Only when iron metabolism indicators are abnormal, iron preparation can prevent the occurrence and development of iron deficiency and prevent the adverse effects of iron overload on the body influence [17]. Since the research on indicators reflecting the iron metabolism status of athletes and the judgment criteria is still in its infancy, the supplementation of iron preparations lacks pertinence. Therefore, it is more scientific and reasonable to supplement the dosage of iron preparations according to the changes of iron metabolism indicators and compound preparations to promote iron preparations absorption. The application still needs further research [18].

## 3. Research Method and Experiment

### 3.1. Method

Iron deficiency and anemia are the most common nutritional disorders in the world. Iron has active redox properties, and appropriate iron levels meet the needs of normal biological functions of cells [19, 20]. In addition to iron, other trace elements can participate in the composition of antioxidant enzymes on the one hand, and on the other hand, trace elements themselves have antioxidant functions. For example, Se is an important component of oxidized glutathione peroxidase, has the ability to scavenge free radicals, and Se itself has antioxidant properties. Zn and Cu jointly participate in the composition of Cu/ZnSOD, and Zn itself has a direct protective effect on the oxidative damage of cell membrane. In addition, Zn can also protect the cell membrane by producing metallothionein and inhibiting the lipid peroxidation of cadmium. However, excessive metal ions can generate a large number of hydroxyl radicals under the action of the Fenton reaction, and the increase of hydroxyl radicals can cause damage to intracellular proteolipid molecules and DNA and finally induce oxidative stress [21, 22]. The relationship between the body's iron status and oxidative stress status is both closely related and intricate.

### 3.2. Experiment

Exercise increases striatal SOD activity or does not alter striatal antioxidant enzyme activity. The experiment herein employed weaned female rats and fed them an iron deficient diet, a standard iron content diet, and an iron overloaded diet. Except for the different iron content in feeds with different iron content, other feed ingredients including other trace elements were the same. The experiment focuses on the effects of long-term aerobic exercise on iron storage in the cerebral cortex, striatum, medulla oblongata, and midbrain, as well as changes in the content of metal ions (Mn, Zn, Cu, and Ca) and their correlation with iron storage.

All the feeds were produced and provided by Nantong Trofi Feed Technology Co. Ltd., and all the nutrients were in accordance with the American Institute of Nutrition (AIN)-93G. In the experiment, various mineral mixtures and vitamin mixtures were created using analytically pure reagents, and mineral and vitamin mixtures were mixed in accordance with AIN-93G to produce finished feeds, which were then expanded into pellet feeds. The iron-deficient dietary feed was formulated according to the basic feed without adding ferric citrate, and the iron content in the iron-deficient feed was controlled to be 12 mg/kg. The iron-overloaded dietary feed was added with 171.1 g of ferric citrate powder on the basis of the basic feed, and the iron content in the iron-overloaded feed was controlled to be 1000 mg/kg. Therefore, in the composition of the three premixes, the remaining components are the same except for the amount of ferric citrate and the amount of fine sucrose.

  SPF healthy Sprague Dawley female rats were randomly divided into 3 groups by random number table method: iron deficiency diet group, normal iron content diet group, and iron overload diet group

The iron-deficient diet group was fed with iron-deficient feed (the iron content in the feed was 12 mg/kg), and the normal iron-content diet group is fed with the standard iron content feed (the iron content in the feed was 45 mg/kg). The iron-overloaded diet group was fed with iron-overloaded feed (the iron content in the feed was 1000 mg/kg). Moreover, the rats were allowed to eat and drink freely, and the drinking water is ultrapure water (resistivity reached 18 MΩ, 25°C). Three weeks after the iron-deficient diet was administered to rats, the plasma iron concentration, blood hemoglobin concentration, and hematocrit all fell, according to observations made before the experiment. Each group was broken into activity and rest groups, including the iron-deficiency diet-exercise group and rest group, the regular iron-content diet-exercise group and rest group, and the iron overload diet-exercise group and rest group. The rats were housed in standard rat cages with stainless steel grid bottoms and in separate cages. There was no difference in food intake between the different groups observed in the pre-experiment and this experiment, and the daily food intake of each rat was about 20 ± 5 g and deionized water was freely drunk.

  After the 3-month swimming exercise, all rats have fasted for 24 hours after the last exercise and the body weight was then weighed

After anesthesia with sodium pentobarbital at a dose of 45 mg/kg body weight, the abdominal cavity was rapidly opened and blood was collected from the heart using a syringe. After the rats were killed by cervical dislocation, the blood vessels were quickly perfused with normal saline to remove the residual blood in the vessels. Moreover, the whole brain was immediately removed by craniotomy, and the brain regions, including the cerebral cortex, striatum, medulla, and midbrain, were rapidly isolated along the midline on the ice surface, taking care to remove superficial blood vessels. At the same time, the liver, spleen, kidney, heart, and other tissues were quickly taken; the fascia, ancillary blood vessels, and fat were removed, and the tissue quality was weighed. After being quick-frozen in liquid nitrogen, it was stored in a −80°C refrigerator for later use.

  The cerebral cortex, striatum, midbrain, medulla oblongata, and spleen tissue (wet) were weighed, and deionized distilled water was added at a ratio of 1 : 10 to make a 10% tissue homogenate in an ice bath

The centrifugation conditions were set to 1500 g and 4°C for 10 min, the precipitate was removed, and the extracted tissue supernatant was centrifuged at 35,000 g and 4°C for 30 min to remove cell debris and organelles, and the supernatant was extracted. Furthermore, the BCA method was used for the determination of soluble protein concentration.

  The content of NHI, Mn, Cu, Zn, Ca, and selenium (Se) was determined by the trichloroacetic acid precipitation method

The tissue homogenate of the sample to be tested was added to the acidic mixture of 0.6 mol/L trichloroacetic acid and was mixed in a water bath at 90°C for 30 min and mixed once every 10 min. Subsequently, centrifugation was performed at 3000 *μ*r/min and 4°C for 5 min. 1.0 mL of the supernatant obtained after centrifugation was accurately aspirated and made up to 10.0 mL with 1% HNO3 solution. The contents of soluble NHI, Mn, Cu, Zn, Ca, and Se in the solution were determined by an inductively coupled plasma mass spectrometer (ICP-MS), and a blank test was also performed. The content of tissue elements was expressed by the content of soluble elements per unit of soluble protein.

MDA content, total SOD activity, RSC, and TAOC assay kits were produced by Nanjing Jiancheng Bioengineering Co. Ltd. The determination of MDA content in the cerebral cortex and striatum tissue homogenate is mainly based on the reaction between MDA and thiobarbituric acid to generate a red compound with a maximum absorption peak at 532 nm. Briefly, 60 *μ*L of supernatant, 60 *μ*L of ultrapure water (as a blank control tube), 60 *μ*L of 10 nMtetraethoxypropane (standard), and 60 *μ*L of anhydrous ethanol solution (standard blank) were sequentially added to the following reactions: (1) 60 *μ*L of trichloroacetic acid-hydrochloric acid solution; (2) 600 *μ*L of 0.1 M hydrochloric acid and 300 *μ*L of 1% thiobarbituric acid; (3) 300 *μ*L of butanol. The above-given mixture was thoroughly mixed and then placed in a water bath at 37°C. for 40 minutes, cooled after the water bath, and centrifuged at 1500 g for 10 minutes. Subsequently, the absorbance value of the supernatant at 532 nm was measured by a microplate reader, and the reference wavelength was 650 nm.

## 4. Result

The effect of dietary iron content on the content of metal ions in the cerebral cortex of female rats is shown in Table 1.

The effect of dietary iron content on striatal metal ion content is shown in Table 2. The results showed that dietary iron deficiency caused a significant increase in striatal Mn content in rats, and dietary iron overload caused a significant increase in striatal NHI content in rats.

The effect of dietary iron content on the content of metal ions in the midbrain are shown in Table 3. The results showed that dietary iron overload caused a significant increase in midbrain NHI content in rats.

The effect of dietary iron content on medulla oblongata metal ion content is shown in Table 4. The results showed that dietary iron deficiency causes significant increases in the contents of NHI, Mn, and Cu in the medulla oblongata of rats, and dietary iron overload causes a significant increase in the contents of NHI and Mn in the medulla oblongata of rats.

As shown in Figure 1, the comparison between LSD groups showed that compared with the corresponding diet resting group, there were no significant differences in the content of NHI, Mn, Cu, Zn, and Ca in the cerebral cortex of IDDE, IADE, and IODE groups (*P* > 0.05). Compared with the corresponding diet resting group, the Se content in the cerebral cortex of the IODE group was significantly increased (*P* < 0.01), and there was no significant difference in the cerebral cortex Se content between the IDDE and IADE groups (*P* > 0.05).

As shown in Figure 2, the comparison between the LSD groups showed that there was no significant difference in striatal NHI content between the IDDE, IADE, and IODE groups compared with the corresponding diet resting group (*P* > 0.05). The striatal Mn content, Cu content, Zn content, and Ca content of IDDE were significantly decreased (*P* < 0.05), but there was no significant difference in striatal Mn content, Cu content, Zn content, and Ca content between IADE and IODE groups (*P* > 0.05).

As shown in Figure 3, the comparison between LSD groups showed that compared with the corresponding diet resting group, the content of NHI in the brain of the IODE group was significantly decreased (*P* < 0.05), and there was no significant difference in the content of NHI in the brain between the IDDE and IADE groups (*P* > 0.05). The brain Cu content in the IADE group was significantly decreased (*P* < 0.05), but there was no significant difference between the IDDE and IODE groups (*P* > 0.05). Moreover, the content of brain Ca in the IODE group was significantly decreased (*P* < 0.05), and there was no significant difference in the content of brain Ca in the IDDE and IADE groups (*P* > 0.05). In addition, there was no significant difference in brain Mn content and Zn content between IDDE, IADE, and IODE groups (*P* > 0.05).

As shown in Figure 4, the comparison between the LSD groups show that compared with the corresponding diet resting group, the content of NHI, Mn, and Cu in the medulla oblongata of the IADE group were significantly increased (*P* < 0.05), while there is no significant difference in the content of NHI, Mn, and Cu in the medulla oblongata of the IDDE and IODE groups (*P* < 0.05). The content of Ca in the medulla of IDDE is significantly decreased (*P* < 0.05), and there is no significant difference in the content of Ca in the medulla of IADE and IODE groups (*P* > 0.05). There is no significant difference in the content of Zn in the medulla oblongata between IDDE, IADE, and IODE groups (*P* > 0.05).

Table 5 shows that the content of MDA in the cerebral cortex of the IDDS group was significantly higher than that of the IADS group (*P* < 0.05). Although the total SOD activity, RSC, and TAOC of the cerebral cortex in the IDDS group are higher than those in the IADS group, there was no significant difference between the two groups (*P* > 0.05). The total SOD activity of the cerebral cortex in the IODS group is higher than that in the IADS group, and the RSC and TAOC were lower than those in the IADS group, but there was no significant difference between the two groups (*P* > 0.05). The results show that the iron-deficient diet causes a significant increase in MDA content in the cerebral cortex of rats.

Table 6 shows that there are no significant differences in striatal MDA content, RSC, total SOD activity, and TAOC in the IODS group compared with the IADS group. The striatal RSC of the IDDS group is significantly lower than that of the IADS group (*P* < 0.001). The results show that an iron-deficient diet causes a significant reduction in striatal RSC in rats.

Table 7 shows that dietary iron content significantly affects TAOC in rat cerebral cortex (*P* < 0.05), but has no significant effect on MDA content, total SOD activity, and RSC in the cerebral cortex (*P* > 0.05). Moreover, exercise factors significantly affect RSC (*P* < 0.001) and TAOC (*P* < 0.05) in the cerebral cortex but have no significant effect on MDA content and total SOD activity in the cerebral cortex (*P* > 0.05). The interaction analysis shows that dietary iron content and exercise had an interaction effect on the MDA content (*P* < 0.01) and total SOD activity (*P* < 0.05) in the cerebral cortex but have no interaction on the RSC and TAOC in the cerebral cortex (*P* > 0.05).

Table 8 shows that the dietary iron content factor significantly affects the striatal RSC of rats (*P* < 0.001) but has no significant effect on the striatal MDA content, total SOD activity, and TAOC (*P* > 0.05). Moreover, exercise factors significantly affect striatal total SOD activity (*P* < 0.05), RSC (*P* < 0.05), and TAOC (*P* < 0.01) but have no significant effect on striatal MDA content (*P* > 0.05). Interaction analysis showed that dietary iron content and exercise have an interaction effect on total SOD activity and RSC in the striatum (*P* < 0.05) but have no interaction effect on striatal MDA content and TAOC (*P* > 0.05).

## 5. Conclusion

In the exercising population, the incidence of iron deficiency and anemia is higher than in the general population, and exercise can alter the iron status in the brain; the maintenance of brain iron homeostasis is essential for the regular functioning of the brain. Consequently, the significance of brain iron in brain function during exercise and the regulation mechanism of brain iron homeostasis will continue to be crucial areas of study in the future.

Additional research at the cellular level will be required in future studies. For instance, starting from the intake of iron to conduct various doses of iron supplementation or supplementation of iron promoters and to study the regulation mechanism of iron homeostasis in the brain has important guiding significance for determining the optimal dose of iron supplementation for exercise individuals. Simultaneously, the control mechanism of iron-deficient diets at different ages and iron supplementation in the latter period on brain iron homeostasis is an additional area of research. In this paper, the effects of dietary iron content and exercise on iron storage, Mn, Cu, and Zn content, and redox state in the brain have been the subject of several theoretical investigations and advances.

## Figures and Tables

**Figure 1:** The effect of exercise under different iron content diets on the content of metal ions in the cerebral cortex of female rats.

**Figure 2:** The effect of exercise on the content of striatal metal ions in rats with different iron content diets.

**Figure 3:** The effect of exercise under diets with different iron contents on the content of metal ions in the midbrain of female rats.

**Figure 4:** The effect of exercise under different iron content diets on the content of metal ions in the medulla oblongata of female rats.

**Table 1:** The effect of dietary iron content on the content of metal ions in the cerebral cortex of female rats.

Group	IDDS	IADS	IODS
NHI (*μ*g/mgpro)	0.13 ± 0.04	0.14 ± 0.04	0.16 ± 0.05
Mn (ng/mgpro)	8.23 ± 0.93	6.53 ± 1.53	5.47 ± 0.84
Cu (ng/mgpro)	38.81 ± 6.01	40.11 ± 11.31	32.71 ± 5.71
Zn (*μ*g/mgpro)	0.33 ± 0.05	0.32 ± 0.08	0.27 ± 0.06
C (*μ*g/mgpro)	0.17 ± 0.04	0.18 ± 0.05	0.14 ± 0.05
Se (ng/mgpro)	0.67 ± 0.27	0.67 ± 0.22	0.58 ± 0.25

**Table 2:** The effect of dietary iron content on striatal metal ion content.

Group	IDDS	IADS	IODS
NHI (*μ*g/mg pro)	0.09 ± 0.03	0.09 ± 0.02	0.12 ± 0.03
Mn (ng/mg pro)	2.84 ± 0.61	2.38 ± 0.28	2.57 ± 0.32
Cu (ng/mg pro)	18.11 ± 4.62	17.91 ± 1.56	18.61 ± 2.98
Zn (*μ*g/mg pro)	0.12 ± 0.03	0.11 ± 0.02	0.12 ± 0.03
C (*μ*g/mg pro)	0.04 ± 0.02	0.03 ± 0.02	0.02 ± 0.02

**Table 3:** The effect of dietary iron content on midbrain metal ion content.

Group	IDDS	IADS	IODS
NHI (*μ*/mgpro)	0.13 ± 0.05	0.14 ± 0.03	0.17 ± 0.04
Mn (ng/mg pro)	5.32 ± 1.18	4.63 ± 0.61	4.65 ± 0.38
Cu (ng/mg pro)	22.92 ± 4.12	22.51 ± 3.81	21.71 ± 2.11
Zn (*μ*g/mg pro)	0.11 ± 0.03	0.11 ± 0.02	0.11 ± 0.02
C (*μ*g/mg pro)	0.03 ± 0.02	0.03 ± 0.02	0.03 ± 0.02

**Table 4:** The effect of dietary iron content on the content of metal ions in the medulla oblongata of female rats.

Group	IDDS	IADS	IODS
NHI (*μ*/mgpro)	0.14 ± 0.04	0.09 ± 0.03	0.16 ± 0.04
Mn (ng/mg pro)	4.39 ± 0.74	3.09 ± 0.63	4.01 ± 0.93
Cu (ng/mg pro)	20.41 ± 4.01	16.01 ± 2.11	19.01 ± 2.81
Zn (*μ*g/mg pro)	0.09 ± 0.03	0.09 ± 0.02	0.11 ± 0.04
C (*μ*g/mg pro)	0.04 ± 0.02	0.03 ± 0.02	0.03 ± 0.02

**Table 5:** The effect of dietary iron content on the redox state of cerebral cortex in female rats.

Group	IDDS	IADS	IODS
MDA content (nmol/mg pro)	1.72 ± 0.15	1.39 ± 0.28	1.64 ± 0.16
Total SOD activity (U/mg pro)	216.49 ± 19.28	195.28 ± 18.19	202.46 ± 9.63
RSC (U/mg pro)	58.16 ± 6.07	51.96 ± 13.29	50.02 ± 9.99
TAOC (U/mg pro)	1.11 ± 0.21	1.01 ± 0.05	0.89 ± 0.09

**Table 6:** The effect of dietary iron content on redox status of the striatum in female rats.

Group	IDDS	IADS	IODS
MDA content (nmol/mg pro)	0.61 ± 0.13	0.82 ± 0.35	0.99 ± 0.39
Total SOD activity (U/mg pro)	261.91 ± 32.29	263.36 ± 55.46	226.05 ± 14.09
RSC (U/mg pro)	45.83 ± 14.88	80.56 ± 11.67	75.37 ± 10.82
TAOC (U/mg pro)	0.86 ± 0.19	0.92 ± 0.12	0.83 ± 0.16

**Table 7:** Two-factor analysis of the effects of dietary iron content and exercise on the redox state of cerebral cortex in female rats.

		Sports	Diet	Exercise × diet
MDA content	*F*	0.58479	0.56762	9.59298
	*P*	0.45753	0.58176	0.00101

Total SOD activity	*F*	1.14231	3.26735	3.48147
	*P*	0.29997	0.05656	0.04747

RSC	*F*	18.78398	1.54833	0.4141
	*P*	0	0.23735	0.67468

TAOC	*F*	6.61247	4.8985	1.71902
	*P*	0.01717	0.01616	0.20402

**Table 8:** Two-factor analysis of the effects of dietary iron content and exercise on redox status of the striatum in female rats.

		Sports	Diet	Exercise × diet
MDA content	*F*	0.2525	2.44622	2.54924
	*P*	0.62721	0.10908	0.101

Total SOD activity	*F*	7.33361	0.13534	4.08343
	*P*	0.01111	0.88375	0.02828

RSC	*F*	5.48531	27.88408	5.31058
	*P*	0.02727	0	0.01111

TAOC	*F*	7.93456	0.03737	0.5858
	*P*	0.00909	0.97364	0.57267

## Data Availability

The data used to support the findings of this study are available from the author upon request.
